The article "Effects of Ziyin Qianyang Formula on Renal Fibrosis through the TGF-β1/Smads Signaling Pathway in Spontaneously Hypertensive Rats" was published in 2022. Journal: Evid Based Complement Alternat Med.

# Effects of Ziyin Qianyang Formula on Renal Fibrosis through the TGF-*β*1/Smads Signaling Pathway in Spontaneously Hypertensive Rats

**DOI:** 10.1155/2022/6088673

**Published:** 2022-11-07

**Authors:** Hui Xu, Chao Wang, Ting-ting Song, Yang Liu, Chang-wu Dong

**Affiliations:** ^1^Anhui University of Chinese Medicine, Hefei 230012, China; ^2^The Second Affiliated Hospital of Anhui University of Chinese Medicine, Hefei 230001, China

## Abstract

**Objective:**

The aim of the study is to explore the effects and mechanisms of action of Ziyin Qianyang Formula (ZYQYF) on renal fibrosis in spontaneously hypertensive rats (SHRs).

**Methods:**

Forty SHRs were randomly divided into a model group, Ziyin Qianyang Formula regular-dose and high-dose groups (ZYQYF-R, 20 g/kg; ZYQYF-H, 40 g/kg), and a western medicine group (enalapril 10 mg/kg), and 10 Sprague-Dawley rats were selected as the normal group. The rats received continuous gavage administration for 6 weeks and systolic blood pressure (SBP) measurements were obtained every fortnight. The serum levels of urea, serum creatinine (sCr), and uric acid (UA) were measured; the pathological morphology and collagen content of the kidneys were observed by hematoxylin-eosin (HE) and Masson staining; and the serum Ang II level was measured by an enzyme-linked immunosorbent assay (ELISA). Transforming growth factor (TGF)-*β*1, Smad-2, Smad-3, and Smad-7 protein and mRNA expressions in kidney tissues was evaluated by western blotting and reverse transcription-polymerase chain reaction.

**Results:**

The ZYQYF-H group showed significantly a lower renal weight and renal weight/body weight than the model group. The enalapril and ZYQYF-H groups showed significantly lower SBP than other groups after 6 weeks of administration. The ZYQYF-H group showed better improvement than the ZYQYF-R and enalapril groups in glomerular and tubular morphology and better reductions in inflammatory cell infiltration and collagen volumetric fraction. The ZYQYF-H group also showed better reductions in serum UA and Ang II levels; collagen-I, collagen-III, and p-Smad2/Smad-2 protein expression; and Smad-2 mRNA expression and a better increase in Smad-7 protein and mRNA expression than the enalapril group. Besides, the degree of renal function and fibrosis improvement was positively correlated with the dose of ZYQYF.

**Conclusion:**

ZYQYF can significantly reduce SHR blood pressure, protect renal function and structure, and improve renal fibrosis by regulating Smad proteins through TGF-*β*1.

## 1. Introduction

Essential hypertension (EH) is a widespread disease of the cardiovascular system and is mainly characterized by an increase in arterial pressure [1]. Despite the availability of various therapeutic agents for hypertension, the incidence of this disease has continued to increase; the number of people with hypertension is expected to grow by 15%–20% each year and reach nearly 1.5 billion patients worldwide by 2025 [2]. Chronic hypertension can cause damage to the kidneys in a variety of conditions and is the second leading cause of end-stage renal disease (ESRD) [3]. Therefore, treatment of hypertension while delaying renal damage is important.

Renal fibrosis is an important pathological manifestation of hypertensive nephropathy [4, 5]. The pathogenesis of hypertensive kidney damage is mainly related to imbalance of extracellular matrix (ECM) production and degradation [6, 7]. Increased activity of the transforming growth factor-*β*1 (TGF-*β*1)/Smads signaling pathway leads to abnormal proliferation and accumulation of fibroblasts in the kidney, and the resultant secretion of large quantities of ECM can cause fibrotic damage in the kidney [8–10]. Our group's previous study showed that Ziyin Qianyang Formula (ZYQYF) had a good antihypertensive effect and could reduce the damage to kidney tissues by regulating the Ang II/TLR4/NF-*κ*B signaling pathway and reducing the expression of inflammatory factors such as interleukin (IL)-6, IL-8, and tumor necrosis factor (TNF)-*α* [11, 12]. However, the effect of this formula on renal fibrosis remains poorly understood. The formula is particularly suitable for patients with “Yin deficiency and Yang hyperactivity” syndrome, which is characterized by the highest serum levels of angiotensin II (Ang II), a powerful factor in inducing the differentiation of periglomerular cells into fibroblasts, among various syndromes [13]. Therefore, the main objective of this study was to investigate the mechanism of action of ZYQYF in improving renal fibrosis in spontaneously hypertensive rats (SHRs) by regulating the Ang II-mediated TGF-*β*1/Smads signaling pathway.

## 2. Materials and Methods

### 2.1. Animals

Forty 12-week-old male SHRs and 10-week-old matched clean-grade Sprague-Dawley (SD) rats weighing 230 ± 10 g were obtained from Beijing Weitong Lihua Experimental Animal Technology Co., Ltd (animal license number SCXK (Beijing): 2016-0011). All rats underwent systolic blood pressure (SBP) measurements after purchase, and SHRs meeting the corresponding blood pressure (SBP > 180 mmHg) criteria were included in the study. These rats were routinely housed at the Animal Experiment Center of Anhui University of Chinese Medicine at a temperature of 20–23°C and humidity of 50%–65%.

### 2.2. Drugs and Reagents

#### 2.2.1. Drugs

The composition of ZYQYF is shown in Table 1. All medicinal herbs used to prepare ZYQYF were purchased from the Second Affiliated Hospital of Anhui University of Chinese Medicine (Anhui, China) and qualified by Professor Dong Chang-wu (Anhui University of Chinese Medicine). All herbs were decocted by an automatic decoction machine. The raw herbs (130 g) were thoroughly washed and soaked in distilled water (1.5 L) for 1 h and then decocted. The extraction solution (0.5 L) was obtained after secondary filtration, equivalent to 0.26 g herbs/mL. Finally, the solution was evaporated to a concentration of 2.0 g herbs/mL (used for ZYQYF-regular-dose) and 4.0 g herbs/mL (used for ZYQYF-high dose) by a rotary evaporator. Enalapril maleate (5 mg/tablet, H32026568, Yisu; Jiangsu Pharmaceutical Co., Ltd., State Drug Administration) tablets were powdered and prepared in a suspension of 1 mg/mL with 0.5% sodium carboxymethyl cellulose (CMC-Na) and stored at 4°C.

#### 2.2.2. Reagents

The reagents obtained for this study were as follows: hematoxylin staining kit (Solarbio, Beijing, China; Lot G1005), Masson staining kit (Solarbio, Beijing, China; Lot G1006), rat Ang II ELISA kit (Elabscience, Wuhan, China; Lot 3PF2QRIH73), collagen-I antibody (Affinity Biosciences, OH, USA; Lot AF7001), collagen-III antibody (Affinity Biosciences, OH, USA; Lot AF5457), TGF-*β*1 antibody (Servicebio, Wuhan, China; Lot GB111876), p-Smad2 antibody (Affinity Biosciences, OH, USA; Lot AF3449), Smad-2 antibody (Servicebio, Wuhan, China; Lot GB11172), p-Smad3 antibody (Cell Signaling Technology, USA; Lot 9523T), Smad-3 antibody (Suzhou Ruiying Biological Co., Ltd, China; Lot RLT4335), Smad-7 antibody (Affinity Biosciences, OH, USA; Lot AF5147), and actin antibody (Servicebio, Wuhan, China; Lot GB12001).

### 2.3. Instruments

The instruments used in this study were as follows: MS60 rat noninvasive blood pressure meter (Shanghai YuYan Scientific Instruments Co., Ltd., China), fully automatic biochemical analyzer (Rayto, Shenzhen, China), RM2016 pathology microtome (Leica, Shanghai, China), Epoch enzyme labeling assay (BioTeK, USA), BV-2 vertical electrophoresis instrument (Servicebio, Wuhan, China), V370 scanner (Seiko Epson Corporation, Japan), KZ-III-FP Grinder (Servicebio, Wuhan, China); CFX Fluorescence Quantitative PCR Instrument (Burroughs), and NanoDrop 2000 Ultra Micro Spectrophotometer (Thermo Fisher Scientific, USA).

### 2.4. Methods

#### 2.4.1. Animal Grouping and Dosing

Ten SD rats were selected as the normal group, while 40 SHRs were randomly divided into the model group, Ziyin Qianyang Formula regular-dose group (ZYQYF-R group), Ziyin Qianyang Formula high-dose group (ZYQYF-H group), and western medicine group (enalapril group; *n* = 10 in each group). On the basis of the adult animal dosages identified in a previous experiment [11], the regular and high doses of ZYQYF were set as 20 and 40 g/kg, respectively. Animals in the western medicine group received enalapril maleate 10 mg/kg by gavage, while those in the normal and model groups received the same volume of CMC-Na by gavage. The rats were gavaged twice a day, at 9: 00 am and 4: 00 pm, for 6 weeks.

#### 2.4.2. Sample Collection

After 6 weeks of gavage and 12 h of fasting, all rats were weighed and anesthetized with pentobarbital sodium 40 mg/kg. Subsequently, 4-5 mL of blood was collected from the abdominal aorta and centrifuged at 3000 r/min and 4°C for 10 min, and the supernatant was separated and stored in a refrigerator at −80°C. After completion of blood collection, the left kidney was quickly obtained, rinsed with saline, dried on filter paper, weighed and divided into two, of which one half was fixed in 4% paraformaldehyde solution and the other half was stored at −80°C in the refrigerator for testing.

### 2.5. Indicator Testing

#### 2.5.1. Blood Pressure Measurement

Using a biosignal acquisition and processing system, a rat pulse transducer was connected to measure the systolic blood pressure in the tail artery. Measurements were taken before and two, four, and six weeks after administration of the drug. Each rat was kept quiet for 30 min; the blood pressure measurements were repeated three times, with a 5-minute interval between each measurement; and the mean value of the measurements was calculated for subsequent analyses.

#### 2.5.2. Measurement of Renal Function Indicators

The serum urea, creatinine (sCr), and uric acid (UA) levels were measured automatically by biochemical analysis instruments.

#### 2.5.3. HE Staining to Observe the Morphological Changes of Kidney Pathology in Each Group of Rats

The left kidney tissue of rats was used to prepare conventional paraffin sections with a thickness of 4 *μ*m. After dewaxing, the sections were stained with hematoxylin for 3 min, rinsed in ultrapure water, stained with eosin solution for 1 min, rinsed with ultrapure water, and then air-dried and sealed with a film. The histopathological morphology of the rat kidney was observed under a light microscope.

#### 2.5.4. Masson Staining of Collagen Fibers in the Kidney Tissue of Rats in Each Group

Paraffin sections were dewaxed with water, stained with iron hematoxylin for 5–10 min, divided using ethanol fractionation, washed once with water, stained in Masson blue solution, and then washed with water. The sections were then stained with acidic Lichon red line red dip for 5–10 min; washed with a weak acid working solution for 1 min; washed in phosphomolybdic acid solution for 1–2 min; washed in a weak acid working solution for 1 min; stained with aniline blue staining solution for 1–2 min; washed with weak acid working solution for 1 min; dehydrated with anhydrous ethanol; and then treated with xylene to make them transparent. The expression of blue-green collagen fibers in rat kidney tissues was observed under a light microscope, and the collagen volumetric fraction (CVF) was analyzed using Image-Pro Plus 6.0 software.

#### 2.5.5. Enzyme-Linked Immunosorbent Assay for the Determination of Ang II in Rat Serum

Frozen serum samples were obtained, and the levels of Ang II in rat serum were determined on the basis of the kit instructions.

#### 2.5.6. Western Blot to Detect the Expression of Collagen-I, Collagen-III, TGF-*β*1, p-Smad2, Smad-2, p-Smad3, Smad-3, and Smad-7 Proteins in Rat Kidney Tissues

After washing 50 mg of rat kidney tissues from each group 2-3 times with PBS, lysis solution equal to 10 times the volume of the tissue was added (protease inhibitor was added a few minutes before use); the sample was then placed on ice and lysed for 30 min, centrifuged for 10 min using a centrifuge at 4°C and 12000 r/min, and the supernatant was obtained to extract the protein. The concentration of the extracted protein was determined using the BCA method. The protein solution was denatured by boiling, electrophoresed, transferred to a membrane, blocked with 5% skimmed milk powder, and phosphorylated proteins were closed with 1% BSA, treated with the primary antibody (1 : 1000 for all objective proteins, 1 : 5000 for internal reference protein) and secondary antibody (1 : 5000) in parallel, incubated and then developed in ECL, decolorized in PhotoShop, and analyzed by Alpha software for optical density values.

#### 2.5.7. Determination of TGF-*β*1, Smad-2, 3, and 7 mRNA Expressions in Rat Kidney Tissues by Reverse Transcription-Quantitative Polymerase Chain Reaction

Total RNA was extracted from rat kidney tissues by the Trizol method; cDNA was synthesized by reverse transcription; and TGF-*β*1 and Smad-2, 3, and 7 mRNA were amplified by adding the corresponding primers. Using 0.2 mL PCR tubes, three tubes were prepared for each reverse transcription product. The specific reaction system included 7.5 *μ*L of 2 × qPCR Mix, 1.5 *μ*L of upstream and downstream primers, 2.0 *μ*L of the cDNA template, and 4.0 *μ*L of ddH_2_O. The reaction conditions were as follows: 40 cycles of pre-denaturation at 95°C (10 min), denaturation at 95°C for 15 s, and annealing/extension at 60°C for 30 s. The fluorescence signal was collected once for every 0.5°C temperature rise from 65°C to 95°C. Data analysis was performed using the 2^−ΔΔ*Ct*^ method. The primer sequences are listed in Table 2.

### 2.6. Blinding Design

The allocation of animals, execution of the experiments, and data analyses were performed by different personnel. The statistical staff were unaware of the specific groupings and were unblinded after the data statistics were analyzed and evaluated.

### 2.7. Statistical Methods

All data were analyzed using SPSS 19.0 software, and the measurement data were expressed as mean ± standard deviation. Data showing a normal distribution were compared using one-way ANOVA, and the LSD method was used when the variance was the same in the two-way comparison, while Dunnett's T3 method was used when the variance was not the same. Differences were considered statistically significant at *P* < 0.05.

## 3. Results

### 3.1. Effects on Renal Weight and Body Weight

In comparison with the normal group, the model and ZYQYF-R groups showed significantly higher renal weight (*P* < 0.01, *P* < 0.05), significantly lower body weight (*P* < 0.05), and significantly higher renal weight/body weight (RW/BW) (*P* < 0.01). Renal weight and RW/BW in the ZYQYF-H and enalapril groups were significantly lower than those in the model group (*P* < 0.05, *P* < 0.01). RW/BW in the enalapril group was significantly lower than that in the ZYQYF-R group () and showed no significant difference from that in the ZYQYF-H group (*P* > 0.05; Figure 1).

### 3.2. Effects on Systolic Blood Pressure

Before administration, the blood pressure of SHRs in all four groups was significantly higher than that of the rats in the normal group (*P* < 0.01). In comparison with systolic blood pressure in the model group, systolic blood pressure was significantly lower in the ZYQYF-R group after 6 weeks of administration (*P* < 0.01), in the ZYQYF-H group after 4 and 6 weeks of administration (*P* < 0.05, *P* < 0.01), and in the enalapril group after 2, 4, and 6 weeks of administration (*P* < 0.01). After 2 and 4 weeks of administration, the systolic blood pressure in the enalapril group was significantly lower than those in the ZYQYF-R and ZYQYF-H groups (*P* < 0.05, *P* < 0.01). However, after 6 weeks of administration, the systolic blood pressure in the enalapril group was not significantly different from that in the ZYQYF-H group (*P* > 0.05; Figure 2).

### 3.3. Effects on the Serum Levels of Urea, sCr, and UA

The serum UA levels in the ZYQYF-H and enalapril groups were significantly higher than that in the normal group (*P* < 0.01), while the serum urea and sCr levels showed no significant difference (*P* > 0.05). The serum urea, sCr, and UA levels in the ZYQYF-R, ZYQYF-H, and enalapril groups were significantly lower than those in the model group (*P* < 0.05, *P* < 0.01). In comparison with the ZYQYF-R group, serum urea, sCr, and UA levels were significantly lower in the ZYQYF-H and enalapril groups (*P* < 0.05, *P* < 0.01). The decrease in serum UA levels was more significant in the ZYQYF-H group than that in the enalapril group (*P* < 0.01; Figure 3).

### 3.4. Effects on Histopathological Morphology of the Kidney

#### 3.4.1. HE Staining

The normal group showed normal glomerular volume, no obvious atrophy, neatly arranged tubular structures, and no obvious inflammatory cell infiltration in the interstitium. In the model group, the glomerular cyst lumen was enlarged, internal atrophy occurred, the tubular lumen was dilated, the structure was unclear and disorganized, and a large number of inflammatory cells were seen infiltrating the interstitium. The ZYQYF-R and enalapril groups showed different degrees of improvement in glomerular morphology, different degrees of reduction in tubular dilatation, neater alignment, and reduced inflammatory cell infiltration in the interstitium. In the ZYQYF-H group, the glomerular morphology was generally normal; the tubular structure was clear and neatly arranged; and only a few inflammatory cells were seen infiltrating the interstitium.  Figure 4.

#### 3.4.2. Masson Staining

The CVF was significantly higher in all SHR groups in comparison with the normal group (*P* < 0.01). However, the CVF in the ZYQYF-H and enalapril groups was significantly lower than that in the model group (*P* < 0.01, *P* < 0.05). Moreover, the CVF in the ZYQYF-H group was significantly lower than those in the ZYQYF-R and enalapril groups (*P* < 0.01, *P* < 0.05; Figure 5).

### 3.5. Effects on the Serum Level of Ang II

In comparison with the normal group, the four SHR groups showed significantly higher serum Ang II levels (*P* < 0.01). In comparison with the model group, the ZYQYF-R, ZYQYF-H, and enalapril groups showed significantly lower serum Ang II levels (*P* < 0.01). In comparison with the ZYQYF-R group, the ZYQYF-H and enalapril groups showed significantly higher serum Ang II levels (*P* < 0.05, *P* < 0.01). The serum Ang II level in the enalapril group was significantly lower than that in the ZYQYF-H group (*P* < 0.05; Figure 6).

### 3.6. Effects on Collagen-I, Collagen-III, TGF-*β*1, p-Smad2, Smad-2, p-Smad3, Smad-3, and Smad-7 Protein Expressions in Kidney Tissues

Collagen-I and collagen-III protein expressions in all SHR groups were significantly higher than those in the normal group (*P* < 0.01). In comparison with the model group, the three treatment groups showed significantly lower expression levels of these two proteins (*P* < 0.01, *P* < 0.05), while the ZYQYF-H group showed significantly lower expression of these proteins in comparison with the ZYQYF-R and enalapril groups (*P* < 0.01).

In comparison with the normal group, only the ZYQYF-H group showed no significant difference in p-Smad3/Smad-3 protein expression (*P* > 0.05). In comparison with the model group, the ZYQYF-R group showed no significant difference in p-Smad2/Smad-2 and p-Smad3/Smad-3 protein expression (*P* > 0.05), while the ZYQYF-H and enalapril groups showed significantly decreased TGF-*β*1, p-Smad2/Smad-2, and p-Smad3/Smad-3 protein expression (*P* < 0.01, *P* < 0.05) and significantly increased Smad-7 protein expression (*P* < 0.01, *P* < 0.05). p-Smad2/Smad-2 protein expression was significantly decreased (*P* < 0.01) and Smad-7 protein expression was significantly increased () in the ZYQYF-H group in comparison with the enalapril group (Figures 7(a)–7(g)).

### 3.7. Effects on TGF-*β*1, Smad-2, 3, and 7 mRNA Expressions in SHR Kidney Tissues

In comparison with the normal group, TGF-*β*1, Smad-2, and Smad-3 mRNA expressions were all significantly upregulated (*P* < 0.05, *P* < 0.01) and Smad-7 mRNA expression was significantly downregulated (*P* < 0.01) in the ZYQYF-R, ZYQYF-H, and enalapril groups. In comparison with the model group, TGF-*β*1, Smad-2, and Smad-3 mRNA expression was all significantly downregulated in the ZYQYF-H and enalapril groups (*P* < 0.05, *P* < 0.01), while only the Smad-2 mRNA expression was significantly downregulated in the ZYQYF-R group (*P* < 0.01), and Smad-7 mRNA expression was significantly upregulated in all three treatment groups (*P* < 0.01). In comparison with the enalapril group, the Smad-2 mRNA expression was significantly downregulated (*P* < 0.05) and the Smad-7 mRNA expression was significantly upregulated (*P* < 0.01) in the ZYQYF-H group. Figures 8(a)–8(d)).

## 4. Discussion

Early renal impairment in patients with EH is often not clinically evident and the symptoms usually appear only when the renal damage is in the middle-to-late stages [14]. Elevated systolic blood pressure and mean arterial pressure are also the most important risk factors for renal impairment in the elderly [15]. Therefore, clinical management of hypertension is based not only on achieving blood pressure targets but also on the maintenance of target organ function. ZYQYF is composed of six herbs: *Radix rehmanniae*, *Rehmannia glutinosa*, Concha Haliotidis, *Uncaria rhynchophylla*, oyster, and *Polygonum multiflorum* Thumb. From a modern medical point of view, the active ingredients of *Radix rehmanniae* and *Rehmannia glutinosa* can protect kidney tubule epithelioid cells and reduce serum urea nitrogen levels [16–18]. Concha Haliotidis can exert a hypotensive effect by influencing the calcium channels and the expression of plasma membrane calcium ATPase (PMCA) mRNA [19]. *Uncaria rhynchophylla* (UR) is known to have significant hypotensive effects and can attenuate Ang II-induced myocardial fibrosis by inhibiting the RhoA/ROCK1 signaling pathway [20]. The oyster extract exhibits antihypertensive effects by inhibiting angiotensin-converting enzyme (ACE) and improves organ inflammation, fibrosis, and apoptosis [21, 22]. Tetrahydroxystilbene glucoside (TSG) is the main active component of *Polygonum multiflorum* Thumb, and it can protect the kidney by inhibiting oxidative stress and reducing inflammatory responses [23]. According to the theory of Chinese medicine, ZYQYF is utilized for “Zi Yin Bu Shen (nourishing Yin and strengthening the kidney)” and “Ping Gan Qian Yang (repressing hyperactive Liver Yang).” The formula thus takes into account both the symptoms and root cause, allowing the smooth reduction of blood pressure and protecting renal function.

These results indicate that a decrease in body weight and an increase in renal weight in the SHR model group in comparison with the SD rats, an alteration that may be related to fibrosis of the kidneys, and that high doses of ZYQYF could alleviate these changes. SHRs typically develop hypertension at 4–6 weeks and gradually show features of hypertensive end-organ damage [24]. The 12-week-old SHRs used in this experiment had significantly elevated blood pressure, elevated related renal function parameters, and pathological changes caused by renal damage, indicating that the animal model is consistent with the typical features of hypertensive renal damage. The results of this study showed no significant decrease in systolic blood pressure in the ZYQYF-R and ZYQYF-H groups after 2 weeks of administration, although a significant decrease in systolic blood pressure was observed in both groups after 6 weeks of administration. Thus, ZYQYF has a definite antihypertensive effect and the accumulation of this effect is needed over time. The systolic blood pressure in the ZYQYF-H group was significantly lower than that in the ZYQYF-R group after 6 weeks of administration, indicating that the antihypertensive effect of ZYQYF was positively correlated with the concentration of the drug administered.

Urea is a sensitive indicator of glomerular filtration function and is often used to assess the degree of progression of renal disease [25]. sCr is also often used in clinical practice to assess the glomerular filtration rate [26]. Elevated serum levels of UA may lead to increased blood pressure through renal inflammation, activation of the renin-angiotensin-aldosterone system (RAAS), and downregulation of NO production, so serum UA levels are closely related to the regulatory system of the kidney [27]. Therefore, the serum levels of urea, creatinine, and UA are important indicators of the renal function. The results of this study showed that ZYQYF significantly reduced the levels of urea, sCr, and UA in SHRs, and the degree of reduction was more obvious in the ZYQYF-H group than in the ZYQYF-R group, with the serum urea and sCr levels in the ZYQYF-H group close to those in normal rats. This finding suggested that ZYQYF could effectively improve the renal function impairment of SHR and the degree of renal function improvement was positively correlated with dose. The results also suggested that ZYQYF can reduce serum UA levels more effectively than enalapril. In addition, the results of HE and Masson staining in this test showed that ZYQYF significantly improved the pathological morphology of glomeruli and tubules in rats and reduced interstitial inflammatory cell infiltration and collagen fiber deposition between tubular interstitial cells, suggesting that ZYQYF not only improved renal function but also had a protective effect on structural aspects of the kidney.

Ang II, an important effector regulated by RAAS, is one of the main mediators in the pathogenesis of EH. On the one hand, Ang II can act directly on the RAAS, stimulating the synthesis of cortisol, regulating the secretion of aldosterone and water and sodium reabsorption, and causing an increase in blood pressure [28]. On the other hand, it regulates the expression of TGF-*β*1 by inducing multiple pathways, which in turn regulates the TGF-*β*1/Smads signaling pathway-mediated renal fibrosis [29]. As seen in the experimental results, ZYQYF can significantly reduce the levels of collagen-I and collagen-III, indicating an improvement in the degree of renal fibrosis. TGF-*β*1 has a strong fibrogenic effect; it can lead to an imbalance om ECM production and degradation and induce proliferation and migration of renal fibroblasts, and its level significantly correlates with the progression of renal interstitial fibrosis [30]. Smad-2, Smad-3, and Smad-7 are the main substrates in the regulation of TGF-*β*1, of which Smad-2 and Smad 3 are receptor-regulated proteins and Smad-7 is an inhibitory protein. In the main process of TGF-*β*1/Smads regulation, the activation of TGF-*β*1 induces phosphorylation of Smad-2 and Smad-3, and the phosphorylated Smad-2 and Smad-3 bind to Smad-4 and signal into the nucleus, thus exerting the effects of cell proliferation, differentiation, apoptosis, and fibrosis. Smad-7 mediates the negative regulatory mechanism of this pathway, regulating the stability of TGF-*β*1 by binding directly to Smads and inhibiting the activity of this pathway [31, 32]. The results of the present study showed that ZYQYF can significantly reduce the serum Ang II level, thereby reducing the activation of the TGF-*β*1/Smads signaling pathway induced by it. Additionally, the results of this study also showed that ZYQYF could effectively inhibit the expression of TGF-*β*1, Smad-2, and Smad-3 proteins and mRNA, and increase the expression of Smad-7 protein and mRNA in kidney tissues, thereby regulating the TGF-*β*1/Smads signaling pathway-mediated renal fibrosis process, and the findings also indicated a dose-effect relationship. On the basis of these findings, ZYQYF can be considered to reduce the degree of renal fibrosis by lowering the serum Ang II level and inhibiting the TGF-*β*1/Smads signaling pathway mediated by Ang II.

## 5. Conclusion

In summary, ZYQYF can significantly reduce systolic blood pressure in SHRs and show good protective effects on both the function and structure of the kidney. Its mechanism of action may involve inhibition of the activation of the Smads signaling pathway, reducing the phosphorylation of Smad-2 and Smad-3, and enhancing the expression of Smad-7 by decreasing the Ang II-mediated expression of TGF-*β*1, which in turn reduces the production of ECM and mitigates the degree of renal fibrosis, playing a role in the treatment of hypertensive renal damage. The present study is limited to the effect of ZYQYF on renal fibrosis through the TGF-*β*1/Smads signaling pathway, but the effect of other signaling pathways and the effect on renal vascular and renal hematological changes require further investigation.

## Figures and Tables

**Figure 1:** Effects on renal weight and body weight. ^△^*P* < 0.05, ^△△^*P* < 0.01 vs. the normal group; ^▲^*P* < 0.05, ^▲▲^*P* < 0.01 vs. the model group; ^*∗*^*P* < 0.05 vs. the ZYQYF-R group. Data are expressed as mean ± SD (*n* = 10). RW/BW: renal weight/body weight.

**Figure 2:** Effects on systolic blood pressure in each group before treatment, 2 weeks after treatment, 4 weeks after treatment, and 6 weeks after treatment. ^△△^*P* < 0.01 vs. the normal group; ^▲^*P* < 0.05, ^▲▲^*P* < 0.01 vs. the model group; ^*∗*^*P* < 0.05, ^*∗∗*^*P* < 0.01 vs. the ZYQYF-R group; ^#^*P*.05, ^##^*P* < 0 < 0.01 vs. the enalapril group. Data are expressed as mean ± SD (*n* = 10).

**Figure 3:** Effects on the serum levels of (a) urea. (b) sCr. (c) UA in each group. ^△△^*P* < 0.01 vs the normal group; ^▲^*P* < 0.05^▲▲^*P* < 0.01 vs. the model group; ^*∗*^*P* < 0.05, ^*∗∗*^*P* < 0.01 vs. the ZYQYF-R group; ^##^*P* < 0.01 vs the enalapril group. Data are expressed as mean ± SD (*n* = 10).

**Figure 4:** Effects on the pathomorphological changes of kidney tissues in various groups of rats (HE, ×200).

**Figure 5:** Effects on the collagen content of kidney tissues in various groups of rats (Masson, ×200). CVF: collagen volumetric fraction, collagen fiber area/total area *∗* 100%.

**Figure 6:** Effects on the serum level of Ang II in each group. ^△△^*P* < 0.01 vs. the normal group; ^▲▲^*P* < 0.01 vs. the model group; ^*∗*^*P* < 0.05, ^*∗∗*^*P* < 0.01 vs. the ZYQYF-R group; ^#^*P* < 0.01 vs. the enalapril group. Data are expressed as mean ± SD (*n* = 10).

**Figure 7:** Effects on collagen-I (b), collagen-III (c), TGF-*β*1 (d), p-Smad2/Smad-2 (e), p-Smad3/Smad-3 (f), and Smad-7 (g) protein expression in the kidney of rats in different groups. ^△^*P* < 0.05, ^△△^*P* < 0.01 vs. the normal group; ^▲^*P* < 0.05, ^▲▲^*P* < 0.01 vs. the model group; ^*∗*^*P* < 0.05, ^*∗∗*^*P* < 0.01 vs. the ZYQYF-R group; ^#^*P* < 0.05, ^##^*P* < 0.01 vs. the enalapril group. Data are expressed as mean ± SD (*n* = 10).

**Figure 8:** Effects on (a) TGF-*β*1. (b) Smad-2. (c) Smad-3. (d) Smad-7 mRNA expression in the kidney of rats of different groups. ^△^*P* < 0.05, ^△△^*P* < 0.01 vs. the normal group; ^▲^*P* < 0.05, ^▲▲^*P* < 0.01 vs. the model group; ^*∗*^*P* < 0.05, ^*∗∗*^*P* < 0.01 vs. the ZYQYF-R group; ^#^*P* < 0.05, ^##^*P* < 0.01 vs. the enalapril group. Data are expressed as mean ± SD (*n* = 10).

**Table 1:** Composition of ZYQYF.

Chinese name	Latin name	Amount (g)
Shengdihuang	*Radix rehmanniae*	15
Shudihuang	*Rehmannia glutinosa*	15
Shijueming	Concha Haliotidis	30
Gouteng	*Uncaria rhynchophylla*	20
Muli	Oyster	30
Heshouwu	*Polygonum multiflorum* thumb	20

**Table 2:** Sequences of primers for PCR.

Gene name	Forward sequence (5′–3′)	Reverse sequence (5′–3′)	Length (bp)
TGF-*β*1	GCTGAACCAAGGAGACGGAATA	GCAGGTGTTGAGCCCTTTCC	194
Smad-2	GTGTCTCATCGGAAAGGGCT	TCATCCAGAGGCGGCAGT	236
Smad-3	TGTCATCTACTGCCGCTTGTG	ATGGCTGTAGTCATCCAGAGGG	220
Smad-7	TCGGAAGTCAAGAGGCTGTGTT	GTTTGAGAAAATCCATCGGGTA	148
GAPDH	CTGGAGAAACCTGCCAAGTATG	GGTGGAAGAATGGGAGTTGCT	138

## Data Availability

The data used to support the findings of this study are available from the first author Hui Xu upon reasonable request.

## Abbreviations

EH: Essential hypertension
ESRD: End-stage renal disease
ECM: Extracellular matrix
TGF-*β*1: Transforming growth factor-*β*1
ZYQYF: Ziyin Qianyang Formula
IL: Interleukin
TNF: Tumor necrosis factor
Ang II: Angiotensin-II
SHR: Spontaneously hypertensive rats
SD: Sprague-Dawley
SBP: Systolic blood pressure
CMC-Na: 0.5% sodium carboxymethyl cellulose
sCr: Serum creatinine
UA: Uric acid
CVF: Collagen volumetric fraction
PMCA: Plasma membrane calcium ATPase
UR: *Uncaria rhynchophylla*
ACE: Angiotensin-converting enzyme
TSG: Tetrahydroxystilbene glucoside
RAAS: Renin-angiotensin-aldosterone system.
